RETRACTED

# Data Mining-Based Analysis of Modern Chinese Medicine for the Treatment of Stable Angina Pectoris in Coronary Heart Disease

**DOI:** 10.1155/2022/3511974

**Published:** 2022-02-28

**Authors:** Min Luo, Yuying Hu, Rong Bai, Zongpei Xu

**Affiliations:** ^1^Graduate School, Tianjin University of Traditional Chinese Medicine, Tianjin 301617, China; ^2^National Clinical Research Center for Chinese Medicine Acupuncture and Moxibustion, First Teaching Hospital of Tianjin University of Traditional Chinese Medicine, Tianjin 300380, China; ^3^Library of Tianjin University of Chinese Medicine, Tianjin University of Traditional Chinese Medicine, Tianjin 301617, China

## Abstract

The aim of this study is to explore the clinical effects of Chinese medicine in the treatment of stable angina pectoris in coronary heart disease. Chinese medicine has multitarget, multilevel, and multilink effects in the treatment of coronary angina, which can significantly improve patients' symptoms. Its mechanism of action involves multiple levels such as regulating lipid metabolism, improving platelet function, antioxidant, and protecting endothelial function. The design was based on data mining to analyse the dosing pattern of modern Chinese medicine for the treatment of stable angina pectoris in coronary heart disease. The number of episodes of angina pectoris, the duration of the episodes, and the changes in the electrocardiogram before and after taking the medicine were observed and compared between the two groups. The number and duration of angina attacks ((2.23 ± 0.77) per week and (1.31 ± 0.34) min/time, respectively) in the study group were found to be significantly better than those in the control group ((3.86 ± 1.03) per week and (2.46 ± 1.21) min/time, respectively).

## 1. Introduction

Coronary atherosclerotic heart disease due to functional changes (stenosis) in the coronary arteries, is collectively known as coronary heart disease [1]. Angina pectoris is a clinical syndrome characterised by chest pain due to temporary myocardial ischaemia and is the most common manifestation of coronary heart disease. The onset of coronary angina is closely related to endothelial dysfunction [2], platelet activation, inflammatory response, plaque rupture, thrombosis, and abnormal serum lipid metabolism. This disease belongs to the category of “chest paralysis and heart pain” in Chinese medicine, and the pathogenesis is “original deficiency and symptomatic deficiency.” Chinese medicine treatment of angina pectoris in coronary artery disease follows the principle of evidence-based treatment and adopts treatment methods such as benefiting Qi, nourishing Yin, invigorating Blood, resolving blood stasis, resolving phlegm, and warming Yang, which has shown certain efficacy advantages [3].

RETRACTED

The duration of angina pectoris is constantly prolonged. Failure to give effective treatment, therefore, tends to allow unstable angina to progress towards acute myocardial infarction [4]. To this end, 63 patients with unstable angina with coronary artery disease who were admitted and diagnosed in this hospital between January 2017 and May 2018 were used as study subjects to explore the clinical effects of Chinese medicine in the treatment of unstable angina with coronary artery disease, with the aim of providing a more accurate and effective Chinese medicine treatment for unstable angina with coronary artery disease[5].

Unstable angina pectoris is unique in its pathophysiological mechanism and therefore requires a robust and aggressive therapeutic intervention in its prevention and treatment [6]. Modern medicine believes that unstable angina is caused by the rupture of arterial plaque and thrombosis, and treatment is usually with anticoagulant, antiplatelet, calcium antagonist, and other thrombolytic drugs; patients with severe symptoms tend to be treated surgically, but the medical costs and risks of Western drugs and surgery are relatively high, and Western drugs focus on a single condition and produce more adverse effects [7, 8]. According to the theory of Chinese medicine, the causes of unstable angina pectorals are many and closely related to the patient's body, such as old age and physical decline, disorders of the internal organs, and poor diet, which can lead to Qi stagnation, blood stasis, and internal phlegm, which can block the veins and block the channels, resulting in chest paralysis and damage to the myocardium to form angina pectoris [9]. In the case of unstable angina, Chinese medicine practitioners often identify the evidence according to the patient's condition, and the method is mostly based on medication, supplemented by acupuncture. According to relevant studies [10], the therapeutic effect of combined Chinese and Western medicine is significantly better than that of single Western medicine. Among the many Chinese medicine prescriptions for the treatment of unstable angina pectoris, Radix Codonopsis bilocular, *Panax notoginseng*, and Radix Panax notoginseng are commonly used. For example, *Astragalus membranaceus* is effective in nourishing Qi and fixing the surface of the body, diuretic, and muscle-building and can be used for hypertension, diabetes, and chronic rhinitis; Radix Codonopsis pilosula is effective in nourishing the middle of the body, strengthening the immune system, enhancing the blood-forming function of the organs, and dilating blood vessels and is effective for spleen deficiency and palpitations; *Panax ginseng* is effective in dispersing blood stasis and stopping bleeding and can be used to treat vomiting of blood, blood in the stool, and stabbing pain in the chest and abdomen; *Salvia metrorrhagia* is effective in promoting pain and activating blood circulation to remove blood stasis. It can remove chest paralysis and relieve heat and pain. Compared with Western medicine, Chinese medicine has better therapeutic effects in the clinical practice of treating unstable angina pectoris in coronary artery disease and reducing the number of angina attacks, which are worthy of clinical promotion.

RETRACTED

## 2. Chinese Medicine in the Treatment of Coronary Heart Disease

The action of TCM in treating diseases is achieved through a multisite, multitarget, and multilevel mechanism of holistic regulation, which in turn is achieved through different combinations of TCM.

### 2.1. Modern Pharmacological Studies on the Active Ingredients of Single-Flavoured Chinese Medicines

*Astragalus*, commonly used as a treatment for angina pectoris in coronary artery disease [11], improves the environment to which blood vessels are exposed, reduces chronic inflammatory cell infiltration, and causes a significant decrease in serum tumour necrosis factor *α*, interleukin 1-beta, and interleukin 6 levels. Meanwhile, the main components of *Astragalus*, amino acids, flavonoids, and astragalosides, can dilate coronary arteries, improve cardiac function, increase resistance to hypoxia, prevent lipid peroxidation, increase myocardial contractility, and reduce blood viscosity by acting on Na+-K+-ATPase [12].It also has a strong free radical scavenging effect, limiting the damage to myocardial cells and subcellular structures caused by oxygen-free radicals.

The main treatment for angina pectoris in coronary artery disease is herbal medicine that activates blood circulation and resolves blood stasis. Studies [13] have shown that *Salvia miltiorrhiza* is a good slow calcium channel blocker and can prevent the disruption of membrane structure and function under ischaemic and hypoxic conditions. Johannessen et al. [14] used ginseng injection and danshen powder injection to treat 52 cases of angina pectoris in coronary heart disease. Danshen powder injection has the effect of inhibiting platelet aggregation and increasing coronary blood flow. It [15] was found that *Calendula officinalis* could significantly reduce whole blood viscosity, plasma viscosity, red blood cell pressure volume, and fibrinogen in patients with coronary heart disease (*P* < 0.05), in order to improve myocardial microcirculation obstruction, so that myocardial ischaemia and hypoxia could be improved and the therapeutic effect of coronary heart disease could be enhanced. Palmer et al. [16] found that *Ligusticum chuanxiong* had the effect of protecting myocardial mitochondrial NOS activity and lowering NO content (*P* < 0.05) and suggested that *Ligusticum chuanxiong* had a protective effect on myocardial ischaemic injury in rats, the mechanism of which might be to inhibit mitochondrial calcium overload and reduce mitochondrial NOS activity, thereby reducing NO-induced injury, scavenging free radicals, and reducing lipid peroxide production. Amrutiya et al. [17] concluded that six commonly used blood-activating herbs, namely, Radix Paeoniae, *Salvia miltiorrhiza*, Chuanxiong, *Panax notoginseng*, peach kernel, and wine rhubarb, could interfere with the progression of mature plaques in ApoE gene-deficient mice and have certain plaque stabilizing effects, the mechanism of which may be related to the regulation of lipid metabolism and inhibition of inflammatory response and reduction of low-density lipoprotein (LDL-C) in rats with myocardial ischaemia.

RETRACTED

The volatile oil of *Citrus aurantium* has antibacterial effects [18] also indicated that the mechanism of action of *Citrus aurantium* to improve vascular endothelial function, stabilize plaque, and reduce cardiovascular events is unknown and may be related to its hypolipidemic, anti-free radical, and anti-inflammatory effects. The active ingredients of centipede can significantly increase superoxide dismutase (SOD) and nitric oxide (NO) content and significantly reduce malondialdehyde (MDA) in rats with myocardial ischaemia, and the ultrastructure showed a significant reduction in cardiomyocyte damage [19].

### 2.2. The Pharmacological Effects of Chinese Herbal Formulations

In the literature [20], it has been proved that the representative drug Shengve capsule, which has the effect of benefiting Qi and nourishing Yin, can enhance myocardial contraction, dilate coronary arteries, increase coronary blood flow, achieve the effect of benefiting Qi and promoting Yang, moving Qi and blood, helping to cure the root cause, thus reducing the attack of angina pectoris.

Heart Ning tablets can increase coronary blood flow, reduce myocardial oxygen consumption, and antiplatelet aggregation, with higher clinical efficacy than compound Dan Shen tablets. The clinical efficacy of Hemifu Bangyu Tang is higher than that of Fuxiang Dan Shen tablets. It can improve the function of the vascular endothelium, thereby improving the efficacy in unstable angina [21].

Lyketos et al. [22] found that heart-supplementing and activating capsules (leech, panel containing, analogue, and astragalus) have definite free radical scavenging ability and antilipid peroxidation effects and have some reversing and protective effects on ischaemic myocardial injury. Yang et al. [21] found that Fuxin Ling granules (Yu Jin, Chuanxiong, Bai Shao, Gan Song, and Ginseng) have improved lipid and blood rheology, regulated endothelin/nitric oxide balance, increased SOD content, and reduced MDA content, thus improving endothelial function and preventing thrombosis and angina attacks. Qishen Yi Qi drops reduces blood lipids and increases ApoA1 levels, which has a beneficial effect in regulating disorders of blood lipid metabolism in patients with coronary heart disease caused by Qi deficiency and blood stasis, thereby alleviating patients' symptoms and reducing the manifestations of TCM symptoms. Banglore et al. [23] found that Fu Zheng and lipid-reducing capsules (*Curcuma longa*, Leech, Da Huang, San Qi, *Astragalus*, etc.) significantly decreased coagulation factor I, D-dimer, and platelet membrane glycoprotein in patients with coronary artery disease (*P* < 0.05), suggesting that the mechanism of action of Fu Zheng and lipid-reducing capsules may be related to improving microcirculation, inhibiting platelet activation and adjusting the coagulation-fibrinolysis balance.

RETRACTED

Tongxinluo capsules (ginseng, leech, scorpion, turtle shell, cicada shed, red peony, and ice chips) have the effects of benefiting Qi, activating blood circulation, relieving spasm and pain, significantly inhibiting inflammation and reducing the levels of hs-CRP, tumour necrosis factor-*α* (TNF-*α*). It also improves the clinical symptoms and electrocardiogram of patients with intractable angina pectoris who have failed to respond to conventional drug therapy. Musk heart pill (musk, sophora, ice chips, ginseng, toadstool, and nux vomica) has the ability to dilate the coronary arteries, increase coronary flow, increase cardiac output, strengthen the heart, resist myocardial ischaemia, protect the myocardium, and scavenge oxygen radicals and is more effective than nitrates in long-term use.

## 3. Analysis of Drug Therapy for Coronary Heart Disease

Based on discrete coronary heart disease, a quantitative coronary heart disease development degree is proposed to characterise the relative levels of different coronary heart disease development by constructing central coronary heart disease and hollow coronary heart disease, which represent the two extremes of positive and negative coronary heart disease.

In this paper, the TOPSIS (Technique for Order Preference by Similarity to an Ideal Solution) method is used to evaluate the degree of development of coronary heart disease. Firstly, a standardised evaluation matrix of coronary heart disease development was developed in the form of $\bar{E}={\left[\bar{e_{ij}}\right]}_{m\times n}$, where *i* is the number of coronary heart diseases to be evaluated, *x*_*i*_ is the number of coronary heart diseases, and *e*_*ij*_ represents the value of the first coronary heart disease for the first developmental characteristic. The standardisation process for cost-based (mobility and energy efficiency) and efficiency-based (size, growth, and balance) characteristics is shown as

(1) $$\begin{array}{c} \bar{e_{ij}}=\frac{\left(\max_{i}e_{ij}-e_{ij}\right)}{\left(\max_{i}e_{ij}-\min_{i}e_{ij}\right)}, \end{array}$$

(2) $$\begin{array}{c} \bar{e_{ij}}=\frac{\left(e_{ij}-\min_{i}e_{ij}\right)}{\left(\max_{i}e_{ij}-\min_{i}e_{ij}\right)}. \end{array}$$

Secondly, the standard deviation method was used to calculate the weights of each developmental feature. If the standard deviation of the *j*th characteristic is *σ*_*j*_, then, the weight of the *n*th developmental characteristic is as follows:

(3) $$\begin{array}{c} w_{j}=\frac{\sigma_{j}}{\sum_{j=1}^{n}\sigma_{j}}. \end{array}$$

Further, the standardised evaluation matrix was weighted to obtain *Z*=[*z*_*ij*_]_*m*×*n*_, of which *z*_*ij*_=*e*_*ij*_ × *w*_*j*_. The maximum value of each development characteristic was used to construct a positive ideal solution of *Z*^+^=[*z*_1_^+^, *z*_2_^+^,…, *z*_*n*_^+^] (*z*_*j*_^+^=max_*i*_*z*_*ij*_), representing a hollow coronary with the greatest potential for electricity load growth. Similarly, a negative ideal solution of *Z*^−^=[*z*_1_^−^, *z*_2_^−^,…, *z*_*n*_^−^] (*z*_*j*_^−^=max_*i*_*z*_*ij*_) was constructed to represent a hollow coronary with less potential for electricity consumption.

RETRACTED

Finally, the degree of coronary heart disease progression is defined as

(4) $$\begin{array}{c} \left\{\begin{array}{c} D_{i}=\frac{{\sqrt{i}}^{-}}{d_{i}^{+}},\\ d_{i}^{+}=\sqrt{\sum_{j=1}^{n}{\left(z_{ij}-z_{j}^{+}\right)}^{2}},\;i=1,2,\ldots ,m,\\ d_{i}^{-}=\sqrt{\sum_{j=1}^{n}{\left(z_{ij}-z_{j}^{-}\right)}^{2}}, \end{array}\right. \end{array}$$

where *d*_*i*_^+^ and *d*_*i*_^−^ are the Euclidean distances of each coronary heart disease from central and hollow coronary heart disease, respectively.

It can be seen that the more developed the coronary heart disease is, the more it tends to be central, and the more likely it is that the implementation of grid construction investment will drive load growth. The less developed coronary heart disease has a significant hollowing out.

*Coronary heart disease data potential curves and the classification of consumption potential types*. First, the data potential ECP can be defined according to a weighted standard evaluation matrix as in equation (5), which quantifies the potential size or level of coronary heart disease data determined by a combination of development characteristics.

(5) $$\begin{array}{c} {\text{ECP}}_{i}=\sum_{j=1}^{n}z_{ij},\;i=1,2,\ldots ,m. \end{array}$$

Further, based on the growth curve function as in (6), the degree of coronary heart disease progression and the corresponding data potential data were fitted to produce a data potential curve.

(6) $$\begin{array}{c} {\text{ECP}}_{i}=\frac{1}{\alpha +\beta e^{-\gamma D_{i}}}. \end{array}$$

By identifying the inflection points above and below the data potential curve, the different types of coronary data potential can be classified as

(7) $$\begin{array}{c} \left\{\begin{array}{cc} \text{Central type,} & D_{i}\geq D_{u},\\ \text{Growth type,} & D_{l}\leq D_{i}<D_{u},\\ \text{Atlanto subtractive type,} & D_{i}<D_{l}. \end{array}\right. \end{array}$$

RETRACTED

## 4. Case Studies

Sixty-three patients with unstable angina pectoris of coronary heart disease admitted and diagnosed in the hospital were selected and divided into two groups according to different treatment methods. The ethics committee of the hospital examined the patients, informed their families, communicated and negotiated, and signed a family notification form. In the control group, there were 32 cases; sex: 18 males and 14 females; and age: 40–67 years, average (60.3 ± 12.5) years. In the study group, there were 31 cases; sex: 17 males and 14 females; age: 42–69 years, mean (62.7 ± 10.6) years.

### 4.1. Results

When comparing the number and duration of angina attacks in the study group with those in the control group, the difference between the study group and the control group before treatment was not statistically significant (*P* > 0.05). After treatment, the number and duration of angina attacks were (2.23 ± 0.77) episodes/week and (1.31 ± 0.34) min/time, respectively, in the study group, which were significantly better than those in the control group ((3.86 ± 1.03) episodes/week and (2.46 ± 1.21) min/time, respectively) (*P* < 0.05). See Table 1.

When comparing the ∑ST and NST values of the two groups after treatment, the ∑ST and NST values of the study group ((0.51 ± 0.29) and (1.79 ± 0.85), respectively) were significantly better than those of the control group ((0.71 ± 0.32) and (2.53 ± 0.62), respectively), with statistically significant differences (*P* < 0.05), as shown in Table 2.

In this paper, the proposed method was validated using the data from our hospital as an example. Factor analysis was performed on the predictor metavariables for the coronary heart disease data, and the main results are shown in Table 3.

RETRACTED

The fitted data potential curves are shown in Figure 1. The data potential types for coronary heart disease were classified according to the upper and lower inflection points, with 39%, 55%, and 6% for decaying, growing, and central coronary heart disease, respectively.

As shown in Figure 2, the number of angina episodes (2.23 ± 0.77) and duration (1.31 ± 0.34) min/time in the study group were significantly better than those in the control group ((3.86 ± 1.03) and (2.46 ± 1.21) min/time), with statistically significant differences (*t* = 3.354, *t* = 4.645, *P* < 0.05). The ∑ST and NST values of the study group ((0.51 ± 0.29) and (1.79 ± 0.85), respectively) were significantly better than those of the control group ((0.71 ± 0.32) and (2.53 ± 0.62), respectively), and the differences were statistically significant (*t* = 4.561, *t* = 4.235, *P* < 0.05).

## 5. Conclusions

Chinese medicine can act on multiple pathological aspects of angina pectoris in coronary heart disease, significantly improving the accompanying symptoms of patients, with relatively few toxic side effects and suitable for long-term application. The mechanisms of action can be summarised as follows: regulation of lipid metabolism and improvement of platelet function and blood rheology. As related clinical and experimental studies continue to be conducted, the mechanism of action of single herbs and compound preparations in the treatment of angina pectoris in coronary artery disease has been further developed, laying the foundation for further elucidation of the mechanism of action of TCM.

## Figures and Tables

**Figure 1:** Data potential curve.

**Figure 2:** Different dosing patterns.

**Table 1:** Number and duration of angina attacks in the study group and control group.

Group	Before treatment		After treatment	
	Number of angina pectoris attacks (times/week)	Attack time of angina pectoris (min/time)	Number of angina pectoris attacks (times/week)	Attack time of angina pectoris (min/time)
Control group (*n* = 32)	8.21±2.67	7.63±2.33	3.83±1.03	2.46±1.21
Study group (*n* = 31)	8.35±2.54	7.42±2.51	2.23±0.77	1.31±0.34
T value	0.682	0.773	3.354	4.645
*P* value	0.112	0.04	0.001	0.001

**Table 2:** Comparison of ∑ST and NST values in the study and control group.

Group	∑ST/mm		Number of NST/leads	
	Before treatment	After treatment	Before treatment	After treatment
Control group (*n* = 32)	1.03±0.45	0.71±0.32	3.23±1.11	2.53±0.62
Study group (*n* = 31)	1.01±0.51	0.51±0.29	3.41±1.09	1.79±0.85
T value	0.696	4.561	0.792	4.235
*P* value	0.078	0.001	0.12	0.002

**Table 3:** Ideal solutions for coronary artery disease.

	Positive ideal solution	Negative ideal solution	Weight
Scale	0.78	0.105	0.413
Growth	0.649	0.076	0.034
Mobility	0.478	−0.234	0.184
Balance	0.343	0.05	0.226
Energy saving level	0.774	0.1	0.143

RETRACTED

## Data Availability

The datasets used during the current study are available from the corresponding author on reasonable request.
